# Retinal Cone Photoreceptors Require Phosducin-Like Protein 1 for G Protein Complex Assembly and Signaling

**DOI:** 10.1371/journal.pone.0117129

**Published:** 2015-02-06

**Authors:** Christopher M. Tracy, Alexander V. Kolesnikov, Devon R. Blake, Ching-Kang Chen, Wolfgang Baehr, Vladimir J. Kefalov, Barry M. Willardson

**Affiliations:** 1 Department of Chemistry and Biochemistry, Brigham Young University, Provo, Utah, United States of America; 2 Department of Ophthalmology and Visual Sciences, Washington University School of Medicine, St. Louis, Missouri, United States of America; 3 Department of Ophthalmology, Baylor College of Medicine, Houston, Texas, United States of America; 4 Department of Biochemistry and Molecular Biology, Baylor College of Medicine, Houston, Texas, United States of America; 5 Department of Ophthalmology, University of Utah Health Science Center, Salt Lake City, Utah, United States of America; 6 Department of Neurobiology and Anatomy, University of Utah Health Science Center, Salt Lake City, Utah, United States of America; 7 Department of Biology, University of Utah, Salt Lake City, Utah, United States of America; University Zürich, SWITZERLAND

## Abstract

G protein β subunits (Gβ) play essential roles in phototransduction as part of G protein βγ (Gβγ) and regulator of G protein signaling 9 (RGS9)-Gβ_5_ heterodimers. Both are obligate dimers that rely on the cytosolic chaperone CCT and its co-chaperone PhLP1 to form complexes from their nascent polypeptides. The importance of PhLP1 in the assembly process was recently demonstrated *in vivo* in a retinal rod-specific deletion of the *Phlp1* gene. To test whether this is a general mechanism that also applies to other cell types, we disrupted the *Phlp1* gene specifically in mouse cones and measured the effects on G protein expression and cone visual signal transduction. In PhLP1-deficient cones, expression of cone transducin (G_t2_) and RGS9-Gβ_5_ subunits was dramatically reduced, resulting in a 27-fold decrease in sensitivity and a 38-fold delay in cone photoresponse recovery. These results demonstrate the essential role of PhLP1 in cone G protein complex formation. Our findings reveal a common mechanism of Gβγ and RGS9-Gβ_5_ assembly in rods and cones, highlighting the importance of PhLP1 and CCT-mediated Gβ complex formation in G protein signaling.

## Introduction

The rod and cone photoreceptor cells of the retina mediate vertebrate vision. These cell types are designed for light detection under different conditions. Rods are high-sensitivity sensors capable of detecting single photons, while cones are lower-sensitivity sensors with a broader dynamic range and faster response kinetics [1]. The two cell types express different visual pigments, with rods expressing rhodopsin and cones expressing up to three distinct cone opsins. The visual pigments are seven transmembrane receptors that couple to heterotrimeric G proteins to initiate a cascade of molecular events that convert photon absorption by the chromophore 11-*cis*-retinal into a neural response in the retina [2].

Two important components of the visual signaling cascade are the G protein β and γ subunit heterodimer (Gβγ) and the regulator of G protein signaling 9 (RGS9)-G protein β_5_ subunit (Gβ_5_) heterodimer. Gβγ forms the visual G protein transducin heterotrimer (G_t_) by binding the transducin α subunit (Gα_t_) and enhancing receptor-mediated GTP exchange on Gα_t_ [3]. RGS9-Gβ_5_ plays a key role in photoresponse recovery by interacting with Gα_t_-GTP and accelerating GTP hydrolysis [4]. Both complexes are obligate dimers, meaning that neither subunit can achieve a stable native state in the absence of the other [5,6]. As a result, dimer formation must be assisted by the cellular chaperone system.

Research into Gβγ and RGS9-Gβ_5_ assembly has shown that the cytosolic chaperonin containing tailless complex polypeptide 1 (CCT) and its co-chaperone, phosducin-like protein 1 (PhLP1), are required for Gβγ and RGS9-Gβ_5_ dimer formation [7]. However, these studies were all performed in cultured cells, leaving questions about their *in vivo* relevance. To address these questions, the *Phlp1* gene (also abbreviated *Pdcl)* was specifically deleted in mouse retinal rods using Cre recombinase-LoxP recognition sequence (Cre-LoxP) gene targeting [8]. PhLP1 deletion caused a striking loss of both Gβγ and RGS9-Gβ_5_ in rods, resulting in reduced sensitivity, decreased amplification rate and prolonged recovery time in rod photoresponses. These findings demonstrated that PhLP1 is required for Gβγ and RGS9-Gβ_5_ assembly in rods and suggested that this mechanism could be shared in other cell types. To test this possibility, we generated a mouse line in which the *Phlp1* gene was disrupted specifically in cone photoreceptors. Cones express a different Gα_t_ (Gα_t2_) and a different Gβγ pair (Gβ_3_γ_c_) than rods [9–11], and they express the same RGS9-Gβ_5_ dimer but at higher concentration [12]. These differences contribute to the unique cone photoresponse sensitivity and kinetics [13,14]. Thus, this mouse allowed us to test the generality of PhLP1-mediated Gβγ and RGS9-Gβ_5_ assembly in a different cell type with a different Gβγ pair and a unique set of G protein signaling properties. We found that PhLP1 deletion caused a marked reduction in expression of G_t2_ and RGS9-Gβ_5_ complexes in cones, which resulted in a major disruption of cone photoresponses. These findings demonstrate that PhLP1 and CCT-dependent folding and assembly of Gβ subunits into complexes are shared between rods and cones, suggesting that these are general chaperones for Gβ complex formation in neurons.

## Materials and Methods

### Development of cone Phlp1 gene deletion

All experiments with mice were performed in strict accordance with National Institutes of Health policy on animal use and were approved by the Brigham Young University and Washington University Institutional Animal Care and Use Committees (PHS assurance numbers: A3783-01 and A3381-01, respectively). Mice were provided food and water *ad libitum* and were euthanized by CO_2_ asphyxiation followed by cervical dislocation. Generation of the *Phlp1-loxP* mouse (PhLP1^F/F^) was described previously [8]. PhLP1^F/F^ mice were bred with the line expressing Cre-recombinase under control of human red/green (HRGP) pigment gene promoter [15] to achieve conditional knockout of the *Phlp1* gene in cone photoreceptors. The HRGP-Cre transgenic mouse expresses Cre-recombinase in both M and S cones in the mouse [15,16]. The animals were bred to maintain a single heterozygous *Cre* ^*+/-*^ allele, and they are referred to hereafter as PhLP1^F/F^Cre^+^ mice. Genotyping for the *Phlp1* ^*F*^ and *Cre* genes was accomplished by PCR detection of mouse ear clips using primers for *Phlp1* ^*F*^ that flanked the LoxP insertion site in intron 3 (f: 5' GAT CAC TTT GAC TGG GGA ATG ATT TTA GGT 3' and r: 5' GAG GTG GTA AGC AGG TGT ACT GGC TGG TTT 3') [8] and primers for HRGP-Cre within the Cre coding sequence (f: 5'-AGG TGT AGA GAA GGC ACT TAG C-3' and r: 5'-CTA ATC GCC ATC TTC CAG CAG G-3') [15].

To create a mouse line in which the cones were genetically labeled, HRGP-Cre mice were crossed with mice harboring a transgene wherein the expression of enhanced green fluorescent protein (EGFP) is driven by a mouse 5.5 Kb green opsin promoter [17]. The *Phlp1* ^*F*^ allele was then bred in to create a knockout that expressed EGFP in the cones. These animals were also bred to maintain a single EGFP allele and are referred to as *PhLP1* ^*F/F*^ *Cre* ^*+*^ *EGFP* ^*+*^ mice. Genotyping primers were within the EGFP coding sequence (f: 5’-ATG GTG AGC AAG GGC GAG GAG-3’ and r: 5’-TGG CGG ATC TTG AAG TTC ACC TTG-3’).

*PhLP1* ^*F/F*^ *Cre* ^*+*^ mice were also bred with *Gnat1* ^*-/-*^ mice in which the gene for Gα_t1_ was disrupted [18], creating a double knockout *PhLP1* ^*F/F*^ *Cre* ^*+*^ *Gnat1* ^*-/-*^ mouse line. In the absence of Gα_t1_ rod phototransduction is blocked, allowing the effects of cone specific deletion of PhLP1 on cone phototransduction to be measured in the absence of rod signaling. Genotyping primers for *Gnat1* were a forward primer in exon 3 (5’-TAT CCA CCA GGA CGG GTA TTC-3’), and reverse primer in the neomycin gene (5’-GGG AAC TTC CTG ACT AGG GGA GG-3’) that detected the disrupted gene, or a reverse primer in exon 4 (5’-GCG GAG TCA TTG AGC TGG TAT-3’) that detected the wild-type gene.

### Antibodies

The following antibodies were used in this study. Primary antibodies: PhLP1 [19], Gβ_1_ [20], RGS9-1 [21] and cone arrestin [22] were made and characterized as described previously by members of our research team. Gα_t2_ and Gγ_c_ [23] was a generous gift from Dr. Vadim Arshavsky (Duke University). Gα_t1_ and Gγ_1_ (Santa Cruz), Gβ_3_ (Sigma), Gβ_5_ (Proteintech), and cone M-opsin (Millipore) were from commercial sources. Secondary antibodies: FITC-conjugated donkey anti-rabbit (Jackson ImmunoResearch Laboratories), TRITC-conjugated peanut agglutinin (Vector Laboratories), AF555-conjugated goat anti-rabbit (Life Technologies) were all from commercial sources.

### Immunohistochemistry and assessment of photoreceptor degeneration

The expression of PhLP1 and other visual signaling proteins in cone photoreceptors was tested by immunocytochemistry as described [8] with some modifications. Briefly, the superior hemisphere of eyes from 30–40 day-old *PhLP1* ^*F/F*^ *Cre* ^*+*^ and control PhLP1^+/+^Cre^+^ mice were cautery-marked for orientation. The eyes were enucleated under ambient illumination without adaptation and the corneas were cut open to allow access of the fixing agent to the interior of the eye. The eyes were immersion-fixed for 1 hr using freshly prepared 4% paraformaldehyde in 0.1 M phosphate buffer (pH 7.4). Fixing for 1 hr compared to the 2 hr time used previously [8] increased detection of PhLP1 in cones compared to rods. After fixing, the eyes were cryo-protected overnight in 30% sucrose in 0.1 M phosphate buffer. The cornea and lens were then removed, and the eyecups were embedded in optimal cutting temperature (OCT) compound for cryo-sectioning. Cryo-sections of 12 μm were cut through the optic nerve head along the vertical meridian and were placed on superfrost microscope slides. For direct comparison, eyes from wild type and knockout animals were cryo-sectioned from the same block and were on the same slide for labeling and microscopy. For immunohistochemistry, sections were rinsed in 0.1 M phosphate buffer and blocked for 1 hr using either 10% donkey serum or 10% normal goat serum, 0.1% Triton X-100 in 0.1 M phosphate buffer. For RGS9-1 and Gβ5 samples, epitopes were retrieved prior to blocking by treating with 1% SDS for 10 min followed by three 10 min washes with 0.1 M phosphate buffer. Primary antibodies to PhLP1 (1:100 dilution), Gα_t2_, Gβ_3_ (1:200), Gγ_c_ (1:50,) M-opsin (1:50), RGS9-1 (1:100), or Gβ_5_ (1:50) were applied to each group of four sections in a humidified chamber overnight at 4°C. After rinsing in three 10-min phosphate buffer washes, FITC-conjugated secondary antibodies at a 1:200 dilution, AF555-conjugated secondary antibodies at a 1:1000 dilution or TRITC-conjugated peanut agglutinin at a 1:200 dilution were applied for 1–2 hrs at room temperature in a light protected, humidified chamber. The sections were viewed using an Olympus FluoView FV1000 confocal laser-scanning microscope with a 60x, 1.4 numerical aperture oil objective lens and an optical slit setting of < 0.9 μm. Images were taken consistently inferior to the optic nerve of each section. All microscope settings including laser transmissivity, PMT voltage, gain, and offset were identical for each set of +/+ and F/F retinal slices imaged by immunofluorescence in order to directly compare fluorescence intensity.

To aid in proper immunolocalization of signaling proteins that are expressed in both rods and cones (PhLP1, RGS9-1, Gβ_5_), immunohistochemistry experiments were performed on *PhLP* ^*F/F*^ *Cre* ^*+*^ *EGFP* ^*+*^ mice to determine the expression of these proteins in cones. Overlapping EGFP fluorescence and AF555 secondary antibody fluorescence indicated expression of PhLP1, RGS9-1 or Gβ_5_ in cones.

Cryo-sections with intact morphology were used for further analysis to determine cone photoreceptor degeneration by staining with TRITC-conjugated peanut agglutinin (PNA) to determine relative cone size and number in mice of 1 and 9 months of age.

### Determination of retinal protein expression

Whole retina extracts were prepared from eyes of age-matched *PhLP1* ^*F/F*^ *Cre* ^*+*^ mice and controls under ambient illumination. These retinas were harvested and placed in ice-cold RIPA buffer (phosphate buffered saline with 1% NP-40 and 6 μl/mL Sigma Protease inhibitor cocktail). The retinas were then passed through an 18G needle 20 times and a 25G needle 10 times to release the proteins. Extracts were centrifuged at 13,800 rpm for 10 min at 4°C to remove cellular debris. Protein concentrations were determined by BCA protein assay, and extracts with equal amounts of protein were resolved on 10% or 14% Tris-glycine-SDS gels or 16.5% Tricine-SDS gels and transferred onto nitrocellulose membranes using an iBlot transfer apparatus (Invitrogen). After blocking with LICOR Blocking buffer for 1 hr, membranes were immunoblotted for each visual protein of interest. The amounts of each protein in the immunoblots were quantified using a LICOR Odyssey near-infrared imaging system and compared to controls.

### Assessment of the photoresponse by electroretinography

Electroretinograms (ERGs) were measured under photopic conditions as follows. One-month old mice were first anesthetized with isofluorane and their pupils were dilated by adding a drop of 1% tropicamide for 15 min to the eyes. A recording electrode was placed on the cornea with a reference electrode inserted subdermally in the cheek and a ground electrode subdermally at the base of the tail. ERG responses were measured using an Ocuscience HMsERG system. Mice were first light adapted for 10 min at a rod-saturating light intensity of 30 cd·s m^˗2^. Full-field photopic ERG recordings of both *PhLP1* ^*F/F*^ *Cre* ^*+*^ and *PhLP1* ^*+/+*^ *Cre* ^*+*^ mice were performed with flashes of increasing white light intensities from 2.3 ×10^–2^ to 1.0 ×10^2^ cd·s m^˗2^ followed by a recovery phase at 30 cd·s m^˗2^. The recovery time between each flash varied from 10 s to 2 min depending on the flash intensities. The amplitudes of the photopic b-wave at different light intensities were then compared between the *PhLP1* ^*F/F*^ *Cre* ^*+*^ and *PhLP1* ^*+/+*^ *Cre* ^*+*^ mice. The intensity–response data were fitted with the Naka–Ruston function [24]: *R = (R*_*max*_ *• I* ^*n*^ *) / (I* ^*n*^ *+ I* ^*n*^_*1/2*_ *)* in which *R* is the transient-peak amplitude of response, *R*_max_ is the maximal response amplitude, *I* is the flash intensity, *n* is the Hill coefficient, and *I*_1/2_ is the half-saturating light intensity. In this case, optimal fits were achieved when the Hill coefficient was set to 1.

ERGs were also measured under scotopic conditions as follows. One-month old mice were dark-adapted overnight and then treated as above without any light adaptation. Full-field scotopic ERG recordings of both *PhLP1* ^*F/F*^ *Cre* ^*+*^ and *PhLP1* ^*+/+*^ *Cre* ^*+*^ mice were performed with flashes of increasing white light intensities from 2.0 ×10^–3^ to 1.0 ×10^2^ cd·s m^-2^. The recovery time of the scotopic ERG between each flash varied from 10 s to 4 min depending on the flash intensities. The amplitudes of the a-wave and b-wave at different light intensities were compared between the *PhLP1* ^*F/F*^ *Cre* ^*+*^ and *PhLP1* ^*+/+*^ *Cre* ^*+*^ mice. The intensity-response data were fitted to a double hyperbolic function [25], again with Hill coefficients set to 1.

### Optomotor responses

*PhLP1* ^*F/F*^ *Cre* ^*+*^ mice were bred with *Gnat1* ^*-/-*^ mice to create a double knockout *PhLP1* ^*F/F*^ *Cre* ^*+*^ *Gnat1* ^*-/-*^ to remove rod signaling that could interfere with cone-driven optomotor responses. Photopic visual acuity and contrast sensitivity of *PhLP1* ^*F/F*^ *Cre* ^*+*^ *Gnat1* ^*-/-*^ and *PhLP1* ^*+/+*^ *Cre* ^*+*^ *Gnat1* ^*-/-*^ mice were measured using a two-alternative forced-choice protocol [26]. The Optomotry system (Cerebral Mechanics) consisted of a square array of four computer monitors with a pedestal in the center where the mouse was placed. A television camera mounted above the animal was used to observe the mouse but not the monitors. Using a staircase paradigm, rotating stimuli (sine-wave vertical gratings) were applied on the monitors where they formed a virtual cylinder around the mouse [27]. The mouse responded to the stimuli by reflexively moving its head in the direction of the rotation. Optomotor responses were measured under photopic background illumination (1.85 log cd m^-2^).

Visual acuity was defined as the threshold for spatial frequency (Fs) of gratings with 100% contrast and measured at the speed (Sp) of 12°/s. At this setting, Fs was gradually increased by the computer protocol until its threshold was determined. Temporal frequency (Ft) was automatically adjusted by the computer program, based on the following equation: Ft = Sp · Fs [26]. Contrast sensitivity was defined as the inverse of contrast threshold for optomotor responses. At this setting, contrast of the stimuli was gradually decreased by the computer protocol until its threshold was determined. Fs was fixed at 0.128 cyc/deg, Ft was set to 1.5 Hz, and Sp was 12°/s. Data were analyzed using independent two-tailed Student's *t*-test, with an accepted significance level of p < 0.05.

### Transretinal ERG recordings

Transretinal ERG recordings were performed as described previously [28]. Briefly, 35–40 day-old *PhLP1* ^*F/F*^ *Cre* ^*+*^ *Gnat1* ^*-/-*^ and *PhLP1* ^*+/+*^ *Cre* ^*+*^ *Gnat1* ^*-/-*^ mice were dark-adapted overnight and then whole retinas were removed from dissected eyecups under infrared illumination. A single retina was placed on the perfusion chamber, between two electrodes connected to a differential amplifier. The retina was perfused with Locke’s solution (112.5 mM NaCl, 3.6 mM KCl, 2.4 mM MgCl_2_, 1.2 mM CaCl_2_, 10 mM HEPES (pH 7.4), 20 mM NaHCO_3_, 3 mM Na succinate, 0.5 mM Na glutamate, 20 μM EDTA, and 10 mM glucose). The perfusion solution was supplemented with 1 mM L-glutamate and 40 μM DL-2-amino-4-phosphonobutyric acid (DL-AP4) to block the postsynaptic components of the photoresponse [29] and 70 μM BaCl_2_ to suppress the slow glial PIII component [30]. The solution was continuously bubbled with a 95% O_2_/5% CO_2_ mixture and heated to 36–37°C. The second retina was stored in oxygenated perfusion solution at room temperature until used, typically within 20–30 min.

Cone-driven responses were recorded using 20 ms test flashes of calibrated 505 nm LED light and its intensity was controlled by an LED-driver and computer in 0.5 log unit steps. Photoresponses were amplified by a differential amplifier (DP-311; Warner Instruments), low-pass filtered at 300 Hz (8-pole Bessel) and digitized at 1 kHz. The intensity-response data were fitted with the Naka-Rushton function as described above, but leaving the Hill coefficient *n* as a variable parameter.

## Results

### Confirmation of PhLP1 deletion in cones

To assess the role of PhLP1 in the assembly of Gβ_3_γ_c_ and RGS9-Gβ_5_ in cone photoreceptors, we created a cone-specific knockout of *Phlp1* by crossing the *PhLP1-loxP* (*Phlp* ^*F/F*^) mouse [8] with the HRGP-Cre mouse in which expression of Cre recombinase in M- and S-cones is driven by the human cone red-green opsin promoter [15,16]. Cre-mediated recombination causes the loss of the translation initiation site of PhLP1, thus removing PhLP1 from cones as soon as the opsins are expressed. Full disruption of the *Phlp1* gene was achieved by generating mice that were homozygous for the *Phlp1* ^*F*^ allele and heterozygous for HRGP-*Cre* allele. The presence of the *Phlp1* ^*F*^ gene was confirmed (Fig. 1A) by a shift in the PCR product (704 bp) compared to the wild type allele (600 bp). PhLP1 protein expression was then tested by immunohistochemistry of PhLP1 in retinal cross-sections. To distinguish PhLP1 expression in cones from that in rods in the photoreceptor layer, we crossed our *PhLP1* ^*F/F*^ *Cre* ^*+*^ mouse line with a mouse line expressing enhanced green fluorescent protein (EGFP) specifically in cones [17] to create a *PhLP1* ^*F/F*^ *Cre* ^*+*^ *EGFP* ^*+*^ mouse line with EGFP-marked cones. Immunolocalization of PhLP1 in these mice showed strong PhLP1 staining in the inner and outer segment of cones with the wild type *Phlp1* allele (*PhLP1* ^*+/+*^ *Cre* ^*+*^ *EGFP* ^*+*^) as evidenced by the co-labeling of the same cones with PhLP1 immunofluorescence (red) and the EGFP fluorescence (green), which was found predominantly in the nuclear region (Fig. 1B). A few PhLP1-labeled cone inner and outer segments showed little EGFP fluorescence because the cell body was out of the confocal plane. In the knockout mice, PhLP1 staining was essentially absent in cones, while background staining in rods and inner retinal cells remained. This result shows that PhLP1 protein expression was specifically lost in the cones of the *PhLP1* ^*F/F*^ *Cre* ^*+*^ *EGFP* ^*+*^ animals.

**Fig 1:** Characterization of the cone photoreceptor-specific PhLP1 knockout mouse. A) PCR genotyping results using the PhLP^F^ primers. The *PhLP1* ^*F*^ gene generated a 704 bp product, while the wild-type gene generated a 600 bp product. B) Immunolocalization of PhLP1 in retinal cross-sections from *PhLP1* ^*+/+*^ *Cre* ^*+*^ *GFP* ^*+*^ and *PhLP* ^*F/F*^ *Cre* ^*+*^ *GFP* ^*+*^ mice expressing EGFP in cones. Immuno-labeling with a PhLP1 primary antibody and AF555-conjugated secondary antibody is shown in red and the EGFP fluorescence is shown in green. These images were merged to show cone expression of PhLP1. C) TRITC-PNA (red) labeling of cones in retinal cross-sections from 1-month and 9-month-old *PhLP* ^*+/+*^ *Cre* ^*+*^ and *PhLP1* ^*F/F*^ *Cre* ^*+*^ mice.

### PhLP1 is not required for cone viability

In rod-specific knockouts, loss of PhLP1 resulted in measurable degeneration of the photoreceptor layer after one month and nearly complete loss of photoreceptors by 6 months [8]. This degeneration was evident by shortening of the photoreceptor outer segments as well as loss of nuclei. To determine if a similar effect would be seen in cone knockouts, we stained cones of one month and nine month old mice with a TRITC-conjugated PNA, which stains the exterior of cone inner and outer segments [31]. *PhLP1* ^*F/F*^ *Cre* ^*+*^ and *PhLP1* ^*+/+*^ *Cre* ^*+*^ mice showed similar number and size of cone cells in both one and nine month old animals (Fig. 1C), indicating that PhLP1deletion did not cause significant cone degeneration up to nine months of age.

### PhLP1 deletion causes a decrease in cone G_t_

Although their overall mechanism for G protein signaling is the same, rods and cones express different G_t_ heterotrimers. Rod photoreceptors use Gα_t1_, Gβ_1_ and Gγ_t1_, whereas cones use Gα_t2_, Gβ_3_ and Gγ_c_. Thus, the deletion of PhLP1 in cones allowed an evaluation of the contribution of PhLP1 to Gβ_3_Gγ_c_ assembly *in vivo*. We first measured the expression of the cone G_t_ subunits in *PhLP1* ^*F/F*^ *Cre* ^*+*^ and *PhLP1* ^*+/+*^ *Cre* ^*+*^ mice by immunohistochemistry. The *PhLP1* ^*F/F*^ *Cre* ^*+*^ mice showed a marked decrease in immuno-labeling of Gα_t2_, Gβ_3_ and Gγ_c_ in the cones (Fig. 2), indicating that expression of the cone G_t_ subunits was substantially reduced. In addition, the residual Gα_t2_ was mislocalized in the absence of PhLP1, with more staining in the cell body and less staining in the outer segment. The effect appeared specific for the cone G_t_ subunits because there was no difference in cone M-opsin expression or localization.

**Fig 2:** Immunolocalization of G_t2_ subunits in PhLP1-deleted cones. A) Retinal cross-sections from *PhLP1* ^*+/+*^ *Cre* ^*+*^ and *PhLP1* ^*F/F*^ *Cre* ^*+*^ mice were probed with antibodies specific to Gα_t2_, Gβ_3_, Gγ_c_, and cone M-opsin and detected with FITC-conjugated secondary antibodies (red).

To further assess the effects of PhLP1 deletion on cone G_t_ expression, whole retina extracts were immunoblotted for cone G_t_ subunits, other cone proteins and rod G_t_ subunits. Gα_t2_ and Gγ_c_ were both reduced significantly in the PhLP1 knockout, while Gβ_3_ was not (Fig. 3). The lack of change in Gβ_3_ expression in whole retina was not unexpected since the PhLP1 deletion was limited to cone cells, and Gβ_3_ is also expressed in other retinal cell types [32,33]. Whole retina expression of PhLP1 itself was consistently decreased by 40% (Fig. 3) despite the fact that there are 30-fold fewer cones than rods in the mouse retina and that PhLP1 is expressed in other retinal cell types [34]. This observation suggests that cones express a higher concentration of PhLP1 than rods and other retinal cells, a finding that is consistent with the intense immuno-labeling of PhLP1 in cones (Fig. 1B). The expression of other cone proteins, M-opsin and cone arrestin, was unchanged in the absence of PhLP1 (Fig. 3B), indicating that the loss of PhLP1 specifically affected cone G_t_ subunit expression and not cone protein expression in general. Rod G_t_ subunit expression was also unchanged, demonstrating that the effect was limited to cones.

**Fig 3:** Protein expression in retina from PhLP1-deleted cones. A) Immunoblots of whole-retinal extracts for PhLP1, cone G_t2_ subunits, RGS9-1, Gβ_5_, M-opsin, cone arrestin, and rod G_t1_ subunits. B) Quantification of immunoblot bands from panel A relative to the wild-type. All data are means ± standard error of the mean (SEM) from 3–6 mice.

### PhLP1 deletion causes a decrease in cone RGS9-Gβ_5_

We previously observed that PhLP1 deletion in rods caused a striking >95% decrease in RGS9-Gβ_5_ expression in those cells, most likely because of an inability to form RGS9-Gβ_5_ dimers [8]. The cone-specific PhLP1 deletion provided an opportunity to test whether this strict PhLP1 dependence for RGS9-Gβ_5_ assembly also applies to cones. To address this question, we measured the effect of PhLP1 deletion on Gβ_5_ and RGS9 expression in cones by immunohistochemistry. We again used EGFP expressing cones to distinguish between cone and rod expression because the extensive Gβ_5_ and RGS9 expression in rods can mask changes in their expression in cones. In the *PhLP1* ^*+/+*^ *Cre* ^*+*^ *EGFP* ^*+*^ control mice, expression of RGS9 was clearly observed in cone outer segments as evidenced by the RGS9 labeling (red) in the outer segments of the EGFP-labeled (green) cones (Fig. 4A). In contrast, the *PhLP1* ^*F/F*^ *Cre* ^*+*^ *EGFP* ^*+*^ knockout mice showed virtually no RGS9 in the outer segments of the EGFP-labeled cones, indicating that RGS9 expression was substantially decreased in PhLP1-deficient cones.

**Fig 4:** Immunolocalization of RGS9-1 and Gβ_5_ in PhLP1-deleted cones. Retinal cross-sections from *PhLP1* ^*+/+*^ *Cre* ^*+*^ and *PhLP1* ^*F/F*^ *Cre* ^*+*^ mice expressing EGFP in cones were probed with antibodies to RGS9 (A) or Gβ_5_ (B) and detected with AF555-conjugated secondary antibody fluorescence (red). EGFP fluorescence (green) marks the cones. The red and green signals were merged to show expression of RGS9 and Gβ5 in cones. White arrows highlight one of several cone outer segments in these views that express RGS9 or Gβ5 and EGFP.

We applied the same strategy to assess Gβ_5_ expression in cones and observed a similar result (Fig. 4B). The number of EGFP-labeled cones with Gβ_5_-labeled outer segments was much less in the PhLP1-deficient cones than in the wild-type cones, indicating expression of Gβ_5_ in cones was impaired in the absence of PhLP1. This decrease in both RGS9 and Gβ_5_ expression in PhLP1-deficient cones argues that RGS9-Gβ_5_ dimer formation is as dependent on PhLP1 in cones as it is in rods. We attempted to confirm the decreased expression by immunoblotting whole retinal extract for Gβ_5_ and RGS9, but saw no differences (Fig. 3B) most likely because the Gβ_5_ and RGS9 expression in rods and the high rod to cone ratio in mouse retina negated our ability to detect their changes in cones.

### PhLP1 knockout results in decreased cone phototransduction

The loss of cone G protein and RGS protein expression would be expected to have a profound effect on phototransduction in cones. To test this possibility, we performed a full-field ERG analysis on *PhLP1* ^*F/F*^ *Cre* ^*+*^ and *PhLP1* ^*+/+*^ *Cre* ^*+*^ mice. Photopic ERG responses, which rely on cone function in bright light, were significantly reduced in *PhLP1* ^*F/F*^ *Cre* ^*+*^ mice compared to control mice, as evidenced by the decreased cone b-wave amplitudes (Fig. 5A). The stimulus-response curve showed a nearly 10-fold decrease in sensitivity, as evidenced by the increased light-intensity required to produce a half-maximal response (I_1/2_) in the PhLP1-deficient animals (Fig. 5C and Table 1). This decrease in sensitivity prevented us from obtaining clearly saturated responses from *PhLP1* ^*F/F*^ *Cre* ^*+*^ cones even with the brightest test flash available in our optical stimulator. However, the estimated maximal response amplitude, R_max_, produced from fitting the data was not statistically different between the two mouse lines (Table 1). In contrast to the reduced sensitivity observed with the photopic responses, scotopic ERG responses, which stem from rod vision under dark-adapted conditions, were essentially identical in the *PhLP1* ^*F/F*^ *Cre* ^*+*^ and *PhLP1* ^*+/+*^ *Cre* ^*+*^ mice (Fig. 5B). The sensitivity and amplitude of both the scotopic a- and b-waves were not different in the knockout mice (Fig. 5D and E), indicating that rod function was unaffected by the cone-specific PhLP1 deletion. These ERG results demonstrate that cone vision is severely impaired in cone-specific PhLP1 knockout mice, as would be expected from the loss of cone G_t_ and RGS9-Gβ_5_ complexes.

**Fig 5:** ERG analysis of cone-specific PhLP1-deleted mice. A-B) Families of ERG responses for *PhLP1* ^*+/+*^ *Cre* ^*+*^ and *PhLP1* ^*F/F*^ *Cre* ^*+*^ mice under photopic (A) and scotopic (B) conditions. Light intensity values are in log candela seconds per square meter. C) Intensity-response relationships for photopic b-waves (n = 8). Data were fit to the Naka-Ruston function that yielded the parameters in Table 1. D-E) Intensity-response relationships for scotopic a-waves (D) and scotopic b-waves (E) (n = 4). Data were fit to a double hyperbolic function (30). All data are means ± SEM.

**Table 1:** ERG parameters for photopic b-waves.

	R_max_ (μV)	I_1/2_ (cd·s·m^-2^)
*PhLP1* ^*+/+*^Cre^+^ (n = 8)	180 ± 3	4.58 ± 0.39
*PhLP1* ^*F/F*^ *Cre* ^*+*^ (n = 9)	168 ± 19 *NS*	39.05 ± 11.42 **

The following parameters are from the fits of the data in Fig. 5C. R_max_, maximal response amplitude

I_1/2_, half-saturating light intensity. Values are means ± SEM. *NS* (not significant) indicates *p* > 0.05 and ** indicates *p* < 0.005, all compared to *PhLP1* ^*+/+*^ *Cre* ^*+*^ values.

To clearly isolate cone photoresponses and overall photopic vision from the dominant rod contribution, we bred the *PhLP1* ^*F/F*^ *Cre* ^*+*^ line onto a Gα_t1_ knockout background (*Gnat1* ^*-/-*^), which removes the Gα_t1_ subunit from rod cells and thus eliminates rod signaling without causing photoreceptor degeneration [35]. These mice were first tested for photopic visual acuity and contrast sensitivity by their optomotor responses to rotating grid stimuli [8]. We found that *PhLP1* ^*F/F*^ *Cre* ^*+*^ *Gnat1* ^*-/-*^ mice had a ~ 2-fold lower visual acuity at the unattenuated luminance level from the computer monitors, as compared to *PhLP1* ^*+/+*^ *Cre* ^*+*^ *Gnat1* ^*-/-*^ animals (Fig. 6A). Moreover, photopic contrast sensitivity of *PhLP1* ^*F/F*^ *Cre* ^*+*^ *Gnat1* ^*-/-*^ animals showed even greater impairment with a nearly 14-fold reduction compared to wild-type (Fig. 6B). These behavioral results further demonstrate that photopic vision is significantly diminished in mice with PhLP1-deficient cones.

**Fig 6:** Visual behavioral and transretinal ERG responses of PhLP1-deficient mice. Photopic visual acuity (A) and contrast sensitivity (B) measurements are shown from *PhLP1* ^*+/+*^ *Cre* ^*+*^ *Gnat1* ^*-/-*^ and *PhLP1* ^*F/F*^ *Cre* ^*+*^ *Gnat1* ^*-/-*^ mice (n = 7 in each group). C-D) Representative families of transretinal cone ERG flash responses from *PhLP1* ^*+/+*^ *Cre* ^*+*^ *Gnat1* ^*-/-*^ (C) and *PhLP1* ^*F/F*^ *Cre* ^*+*^ *Gnat1* ^*-/-*^ (D) mice. Test flashes of increasing intensities were delivered at time 0. The red traces show responses to an intensity of 5.7×10^4^ photons μm^-2^. E) Intensity-response functions for transretinal cone ERG responses from *PhLP1* ^*+/+*^ *Cre* ^*+*^ *Gnat1* ^*-/-*^ (n = 9) and *PhLP1* ^*F/F*^ *Cre* ^*+*^ *Gnat1* ^*-/-*^ (n = 13) mice. Data were fit to the Naka-Ruston function that yielded the parameters in Table 2. F) Amplification of the phototransduction cascade in mouse cones. The rising phases of the light responses were matched for *PhLP1* ^*+/+*^ *Cre* ^*+*^ *Gnat1* ^*-/-*^ at 2.4 x 10^3^ photons μm^-2^ and *PhLP1* ^*F/F*^ *Cre* ^*+*^ *Gnat1* ^*-/-*^ at 5.7 x 10^4^ photons μm^-2^ by down scaling the *PhLP1* ^*F/F*^ *Cre* ^*+*^ *Gnat1* ^*-/-*^ response by a factor of 4.5. The figure shows the match in the rising phase produced by this procedure. A 5.3-fold decrease in amplification constant in the *PhLP1* ^*F/F*^ mice can be calculated from the ratio of the *PhLP1* ^*F/F*^ to *PhLP1* ^*+/+*^ light intensity after correction by the scaling factor. G) Kinetics of cone dim flash responses. Normalized population-averaged dim flash responses to light intensities of 2.4×10^3^ photons μm^-2^ for *PhLP1* ^*+/+*^ *Cre* ^*+*^ *Gnat1* ^*-/-*^ (n = 9) and 5.7×10^4^ photons μm^-2^ for *PhLP1* ^*F/F*^ *Cre* ^*+*^ *Gnat1* ^*-/-*^ (n = 12), demonstrating the decelerated photoresponse recovery in PhLP1-deficient cones. All data are means ± SEM.

**Table 2:** Cone transretinal ERG parameters.

	R_max_ (μV)	T_peak_ (ms)	T_integr._ (ms)	S_f(n)_ (μm^2^/ph)	I_1/2_ (ph/μm^2^)	n (I_1/2_)	τ_rec_ (ms)
*PhLP1* ^*+/+*^Cre^+^ *Gnat1* ^*-/-*^ (n = 9)	50.9 ± 4.1	56.3 ± 1.1	59.9 ± 1.7	6.8x10^–5^ ± 5.2x10^–6^	1.6x10^4^ ± 0.2x10^4^	0.94 ± 0.02	28.9 ± 2.8
*PhLP1* ^*F/F*^Cre^+^ *Gnat1* ^*-/-*^ (n = 12)	43.1 ± 2.9 *NS*	219.8 ± 9.2 ***	1165.3 ± 46.0 ***	2.9x10^–6^ ± 1.7x10^–7^ ***	4.3x10^5^ ± 0.3x10^5^ ***	0.91 ± 0.02 *NS*	1106.9 ± 61.9 ***

The following parameters are from the fits of the data in Fig. 6. R_max_, maximal response amplitude

time-to-peak (T_peak_) and integration time (T_integr._) refer to responses whose amplitudes were < 0.2 R_max_ and fell within the linear range

S_f(n),_ normalized dim flash fractional sensitivity (amplitude of dim flash response divided by flash strength and then normalized for the amplitude of saturating response)

I_1/2_, half-saturating light intensity

n (I_1/2_), Hill coefficient in the Naka-Rushton equation

τ_rec_, time constant of single-exponential decay of dim flash response recovery phase. Values are means ± SEM. *NS* (not significant) indicates *p* > 0.05 and *** indicates *p* < 0.001, all compared to *PhLP* ^*+/+*^ *Cre* ^*+*^ *Gnat1* ^*-/-*^ values.

To investigate the effects of PhLP1 deletion on cone signaling more specifically, we measured cone photoresponses by transretinal ERG recordings from dark-adapted mouse retinas using the same line of animals on the *Gnat1* ^*-/-*^ background. Synaptic inhibitors were used to facilitate cone recordings by blocking post-photoreceptor components of the photoresponse (see Materials and Methods). Similar to the live animal ERG recordings, dark-adapted cones from *PhLP1* ^*F/F*^ *Cre* ^*+*^ *Gnat1* ^*-/-*^ mice showed substantially decreased light sensitivity compared to wild-type controls (Fig. 6 C,D). This phenomenon could be easily seen by comparing the responses at 5.7×10^4^ photons μm^-2^ (Fig. 6C and D, red traces). Stimulus-response curves further illustrated the decreased sensitivity, showing a 27-fold increase in I_1/2_ in the knockout mice (Fig. 6E and Table 2). By comparison, the reduction in cone sensitivity in isolated retinas was three times greater than that seen in the live animal ERG recordings, providing a more accurate measure of the diminished cone sensitivity given that the transretinal ERG recordings measure cone a-wave responses directly, while the live animal ERGs measure subsequent b-wave responses from downstream bipolar neurons. Similar to the *in vivo* ERG, saturated cone responses could not be achieved with the *PhLP1* ^*F/F*^ *Cre* ^*+*^ *Gnat1* ^*-/-*^ mice because of their reduced light sensitivity, but the R_max_ value determined from fitting the data again showed no significant difference from the *PhLP1* ^*+/+*^ *Cre* ^*+*^ *Gnat1* ^*-/-*^ mice (Table 2), further indicating that the number of cones and length of their outer segments were similar in the two mouse lines as observed in the cone morphology data (Fig. 1C).

From the transretinal ERG data, we were able to assess the effect of PhLP1 deletion on the relative cone phototransduction amplification by comparing the intensities of light required to produce identical dim flash response activation phases. We compared population-averaged fractional responses in the linear range that corresponded to 5.7×10^4^ photons μm^-2^ for *PhLP1* ^*F/F*^ *Cre* ^*+*^ *Gnat1* ^*-/-*^ cones, and 2.4×10^3^ photons μm^-2^ for *PhLP1* ^*+/+*^ *Cre* ^*+*^ *Gnat1* ^*-/-*^ cones (Fig. 6F). To match the rising phases, the fractional dim flash *PhLP1* ^*F/F*^ *Cre* ^*+*^ *Gnat1* ^*-/-*^ response required further downscaling by an average factor of 4.5. Thus, the ratio of the two light intensities corrected by the scaling factor yielded a 5.3-fold reduction in the signal amplification in *PhLP1* ^*F/F*^ *Cre* ^*+*^ *Gnat1* ^*-/-*^ cones. This reduction can be explained by the reduced expression and the mislocalization of Gα_t2_ observed in *PhLP1* ^*F/F*^ *Cre* ^*+*^ cones (Fig. 3A, B).

### PhLP1 knockout results in prolonged cone photoresponse recovery

RGS9-Gβ_5_ is highly expressed in cones and is believed to contribute substantially to the rapid photoresponse recovery rate characteristic of cones [12,14,36]. Thus, the loss of RGS9-Gβ_5_ upon PhLP1 deletion (Fig. 2B) would be expected to decelerate the cone response recovery. Indeed, there was a striking delay in the recovery phase of the cone photoresponses accompanied by an unusual biphasic waveform (Fig. 6G). The dim flash recovery time constant (τ_rec_) was increased 38-fold (Table 2), eight times more than was seen upon PhLP1 deletion in rods [8]. This dramatic decrease in the cone response recovery rate is very similar to that observed in RGS9 knockout mice [36] and provides direct evidence that efficient assembly of RGS9-Gβ_5_ complex by PhLP1 plays a key role in the rapid kinetics of dark-adapted cone photoresponses.

## Discussion

### PhLP1 and cone G_t_ function

This study demonstrates the essential role of PhLP1 in mammalian cone physiology by eliminating it specifically in mouse cones. The loss of PhLP1 substantially reduced expression of all three subunits of the cone G_t_ heterotrimer (Figs. 2 and 3), and resulted in a marked desensitization of photopic photoresponses (Figs. 5 and 6). These findings are similar to those of the rod-specific PhLP1 deletion, which also showed reductions in rod G_t_ subunits resulting from an inability to form Gβ_1_γ_1_ heterodimers [8]. Likewise, the observed loss of cone G_t_ can be attributed to an inability to form Gβ_3_γ_c_ dimers in the absence of PhLP1. This observation provides *in vivo* evidence for the hypothesis, developed from studies in cell culture, that all Gβγ dimer combinations require PhLP1 for assembly [37]. The loss of Gβ_3_γ_c_ leads to a reduction in Gα_t2_ and its partial mis-localization from the cone outer segment to the inner segment and cell body (Fig. 2). Interestingly, a recent study of a Gβ_3_ knockout mouse showed a similar mis-localization of Gα_t2_ in the cone inner segment [38], lending further support to the idea that Gβ_3_γ_c_ plays an important role in the localization of Gα_t2_ to the outer segment.

The reduction in cone G_t_ subunits was accompanied by a substantial deterioration in photopic vision, demonstrated by full-field ERG and visual behavioral tests (Figs. 5 and 6A, B). This effect was even greater in transretinal ERG recordings, with a 27-fold decrease in light sensitivity of dark-adapted cones and a 5.3-fold decrease in their signal amplification, when all rod signaling was eliminated by Gα_t1_ deletion (Fig. 6 and Table 2). However, the maximum amplitude of the cone photoresponse was not significantly changed, consistent with our finding that other components of the cone visual cascade such as cone opsins (Fig. 3A, B) remained unaltered in the PhLP1 knockout. These effects on cone phototransduction are similar to those of the Gβ_3_ knockout [38], supporting the idea that formation of functional Gβ_3_γ_c_ dimers was greatly reduced in the absence of PhLP1.

An additional question concerns the source of the residual cone photoresponse in the PhLP1 knockout. The residual photoresponse showed unusual biphasic kinetics that may reflect two populations of cone transducin, a smaller population with near normal activation kinetics and a larger population with greatly reduced activation kinetics. Perhaps the smaller population represents residual intact G_t2_ heterotrimers containing Gβ_3_γ_c_ assembled in the absence of PhLP1, while the larger population represents Gα_t2_ monomers that are activated in the absence of Gβ_3_γ_c_. A growing body of evidence argues that Gα_t_ monomers can be activated by opsins, albeit less efficiently, from both cone photoresponses in a Gβ_3_ knockout [38] and from rod photoresponses in the rod-specific PhLP1 knockout [8] and two Gγ_1_ knockout lines [39,40]. Insight into a possible means of activating Gα_t_ in the absence of Gβγ can be gleaned from the atomic structure of the complex between the G_s_ heterotrimer and an agonist-bound β-adrenergic receptor [41]. In this complex, there were no direct contacts between Gβ_1_γ_2_ and the receptor, but interactions between Gβ_1_ and the N-terminus of Gα_s_ positioned the N-terminus next to the membrane where it made important contacts with the receptor. In the case of Gα_t_ and opsins, the high concentration of Gα_t_ in rod and cone photoreceptors may permit inefficient activation in the absence of these interactions of Gβγ.

### PhLP1 and RGS9-Gβ_5_ assembly in cones

Previous work showed that the deletion of either RGS9 or Gβ_5_ resulted in complete loss of the other in rod cells and lead to the conclusion that RGS9-Gβ_5_ was an obligate dimer [5,21]. Hence, the loss of RGS9 and Gβ_5_ in the cone-specific PhLP1 knockout (Fig. 2B) is indicative of an inability to form RGS9-Gβ_5_ heterodimers. This conclusion is supported by the 38-fold prolongation of cone response shutoff time in the absence of PhLP1 (Fig. 6 and Table 2). This result parallels findings from cones of *RGS9* ^*-/-*^ mice, which showed a 60-fold prolongation of the shut-off time [36]. The similar degree of these effects indicates that RGS9-Gβ_5_ complexes are severely depleted in PhLP1-deficient cones. Thus, our results demonstrate that the assembly of the RGS9-Gβ_5_ complex in cones is critically dependent on PhLP1.

The same loss of both Gβ_5_ and RGS9 in the absence of PhLP1 was also observed in rods [8], although the 5-fold increase in rod shutoff time was less striking [8]. Several studies have shown that cones express higher levels of RGS9-1 and Gβ_5_ than rods, which is believed to contribute to the rapid recovery kinetics of cone responses [12,14]. Perhaps the higher expression of PhLP1 that we observed in cones (Figs. 1 and 3) supports a greater demand for RGS9-Gβ_5_ assembly in cones.

### PhLP1 and cone viability

PhLP1 deletion in mouse rods results in fairly rapid photoreceptor degeneration [8], yet we did not observe a similar degeneration in PhLP1-deficient cones up to 9 months of age (Fig. 1D). It is believed that rod degeneration in the absence of PhLP1 is caused by the accumulation of Gβ_1_ on CCT [8], eventually causing massive chaperone and proteasomal overload and cell death [42]. The lack of degeneration of PhLP1-deficient cones would suggest that their chaperonin system is not as compromised by the loss of PhLP1. One possibility is that Gβ_3_ is more easily cleared from CCT than Gβ_1_. Consistent with this hypothesis, Gβ_3_ has been shown to have lower affinity for CCT than Gβ subunit isoforms 1, 2, and 4 [43]. Alternatively, rod-derived survival factors may maintain cone viability [44,45] despite possible insults to the cone proteome from diminished CCT function in the absence of PhLP1.

In summary, the deletion of PhLP1 in cone photoreceptors results in the loss of cone G_t_ heterotrimers and RGS9-Gβ_5_ dimers and leads to a marked reduction in cone light sensitivity and a greatly retarded photoresponse recovery. These findings parallel those of the PhLP1 deletion in rod photoreceptors [8], demonstrating a common mechanism of Gβγ and RGS9-Gβ_5_ formation in rods and cones. The results predict that PhLP1- and CCT-mediated assembly of these complexes is shared in other neurons, where PhLP1 is also expressed [46], highlighting the general importance of these chaperones in neuronal G protein signaling.

## References

[1] KefalovVJ (2012) Rod and cone visual pigments and phototransduction through pharmacological, genetic, and physiological approaches. J Biol Chem 287: 1635–1641. 10.1074/jbc.R111.303008 22074928PMC3265844

[2] ArshavskyVY, BurnsME (2012) Photoreceptor signaling: supporting vision across a wide range of light intensities. J Biol Chem 287: 1620–1626. 10.1074/jbc.R111.305243 22074925PMC3265842

[3] FungBK-K (1983) Characterization of transducin from bovine retinal rod outer segments. J Biol Chem 258: 10495–10502. 6136509

[4] ArshavskyVY, WenselTG (2013) Timing is everything: GTPase regulation in phototransduction. Invest Ophthalmol Vis Sci 54: 7725–7733. 10.1167/iovs.13-13281 24265205PMC3837634

[5] ChenCK, Eversole-CireP, ZhangH, MancinoV, ChenYJ, et al (2003) Instability of GGL domain-containing RGS proteins in mice lacking the G protein beta-subunit Gbeta5. Proc Natl Acad Sci U S A 100: 6604–6609. 1273888810.1073/pnas.0631825100PMC164494

[6] HigginsJB, CaseyPJ (1994) In vitro processing of recombinant G protein gamma subunits. Requirements for assembly of an active beta gamma complex. J Biol Chem 269: 9067–9073. 8132644

[7] WillardsonBM, TracyCM (2012) Chaperone-mediated assembly of G protein complexes. Subcell Biochem 63: 131–153. 10.1007/978-94-007-4765-4_8 23161137

[8] LaiCW, KolesnikovAV, FrederickJM, BlakeDR, JiangL, et al (2013) Phosducin-Like Protein 1 is Essential for G-Protein Assembly and Signaling in Retinal Rod Photoreceptors. J Neurosci 33: 7941–7951. 10.1523/JNEUROSCI.5001-12.2013 23637185PMC3695707

[9] LeeRH, LiebermanBS, YamaneHK, BokD, FungBK (1992) A third form of the G protein beta subunit. 1. Immunochemical identification and localization to cone photoreceptors. J Biol Chem 267: 24776–24781. 1447215

[10] LereaCL, SomersDE, HurleyJB, KlockIB, Bunt-MilamAH (1986) Identification of specific transducin alpha subunits in retinal rod and cone photoreceptors. Science 234: 77–80. 352939510.1126/science.3529395

[11] OngOC, YamaneHK, PhanKB, FongHK, BokD, et al (1995) Molecular cloning and characterization of the G protein gamma subunit of cone photoreceptors. J Biol Chem 270: 8495–8500. 772174610.1074/jbc.270.15.8495

[12] CowanCW, FarissRN, SokalI, PalczewskiK, WenselTG (1998) High expression levels in cones of RGS9, the predominant GTPase accelerating protein of rods. Proc Natl Acad Sci U S A 95: 5351–5356. 956027910.1073/pnas.95.9.5351PMC20264

[13] NikonovSS, KholodenkoR, LemJ, PughENJr. (2006) Physiological features of the S- and M-cone photoreceptors of wild-type mice from single-cell recordings. J Gen Physiol 127: 359–374. 1656746410.1085/jgp.200609490PMC2151510

[14] ZhangX, WenselTG, KraftTW (2003) GTPase regulators and photoresponses in cones of the eastern chipmunk. J Neurosci 23: 1287–1297. 1259861710.1523/JNEUROSCI.23-04-01287.2003PMC6742256

[15] LeYZ, AshJD, Al-UbaidiMR, ChenY, MaJX, et al (2004) Targeted expression of Cre recombinase to cone photoreceptors in transgenic mice. Mol Vis 10: 1011–1018. 15635292

[16] LeYZ, AshJD, Al-UbaidiMR, ChenY, MaJX, et al (2006) Conditional gene knockout system in cone photoreceptors. Adv Exp Med Biol 572: 173–178. 1724957210.1007/0-387-32442-9_26

[17] ChenFS, ShimH, MorhardtD, DallmanR, KrahnE, et al (2010) Functional redundancy of R7 RGS proteins in ON-bipolar cell dendrites. Invest Ophthalmol Vis Sci 51: 686–693. 10.1167/iovs.09-4084 19797210PMC2868441

[18] CalvertPD, KrasnoperovaNV, LyubarskyAL, IsayamaT, NicoloM, et al (2000) Phototransduction in transgenic mice after targeted deletion of the rod transducin alpha-subunit. Proc Natl Acad Sci USA 97: 13913–13918. 1109574410.1073/pnas.250478897PMC17675

[19] ThulinCD, HowesK, DriscollCD, SavageJR, RandTA, et al (1999) The immunolocalization and divergent roles of phosducin and phosducin-like protein in the retina. Mol Vis 5: 40 10617777

[20] LeeBY, ThulinCD, WillardsonBM (2004) Site-specific phosphorylation of phosducin in intact retina. Dynamics of phosphorylation and effects on G protein beta gamma dimer binding. J Biol Chem 279: 54008–54017. 1548584810.1074/jbc.M405669200

[21] ChenCK, BurnsME, HeW, WenselTG, BaylorDA, et al (2000) Slowed recovery of rod photoresponse in mice lacking the GTPase accelerating protein RGS9-1. Nature 403: 557–560. 1067696510.1038/35000601

[22] ZhangT, BaehrW, FuY (2012) Chemical chaperone TUDCA preserves cone photoreceptors in a mouse model of Leber congenital amaurosis. Invest Ophthalmol Vis Sci 53: 3349–3356. 10.1167/iovs.12-9851 22531707PMC3385966

[23] LobanovaES, HerrmannR, FinkelsteinS, ReidelB, SkibaNP, et al (2010) Mechanistic basis for the failure of cone transducin to translocate: why cones are never blinded by light. J Neurosci 30: 6815–6824. 10.1523/JNEUROSCI.0613-10.2010 20484624PMC2883257

[24] NakaKI, RushtonWA (1966) S-potentials from luminosity units in the retina of fish (Cyprinidae). J Physiol 185: 587–599. 591806010.1113/jphysiol.1966.sp008003PMC1395832

[25] LobanovaES, FinkelsteinS, HerrmannR, ChenYM, KesslerC, et al (2008) Transducin gamma-subunit sets expression levels of alpha- and beta-subunits and is crucial for rod viability. J Neurosci 28: 3510–3520. 10.1523/JNEUROSCI.0338-08.2008 18367617PMC2795350

[26] UminoY, SolessioE, BarlowRB (2008) Speed, spatial, and temporal tuning of rod and cone vision in mouse. J Neurosci 28: 189–198. 10.1523/JNEUROSCI.3551-07.2008 18171936PMC2847259

[27] PruskyGT, AlamNM, BeekmanS, DouglasRM (2004) Rapid quantification of adult and developing mouse spatial vision using a virtual optomotor system. Invest Ophthalmol Vis Sci 45: 4611–4616. 1555747410.1167/iovs.04-0541

[28] KolesnikovAV, KefalovVJ (2012) Transretinal ERG recordings from mouse retina: rod and cone photoresponses. J Vis Exp: e3424.10.3791/3424PMC346059222453300

[29] SillmanAJ, ItoH, TomitaT (1969) Studies on the mass receptor potential of the isolated frog retina. I. General properties of the response. Vision Res 9: 1435–1442. 536743310.1016/0042-6989(69)90059-5

[30] NymarkS, HeikkinenH, HaldinC, DonnerK, KoskelainenA (2005) Light responses and light adaptation in rat retinal rods at different temperatures. J Physiol 567: 923–938. 1603709110.1113/jphysiol.2005.090662PMC1474229

[31] BlanksJC, JohnsonLV (1984) Specific binding of peanut lectin to a class of retinal photoreceptor cells. A species comparison. Invest Ophthalmol Vis Sci 25: 546–557. 6715128

[32] DhingraA, RamakrishnanH, NeinsteinA, FinaME, XuY, et al (2012) Gbeta3 is required for normal light ON responses and synaptic maintenance. J Neurosci 32: 11343–11355. 10.1523/JNEUROSCI.1436-12.2012 22895717PMC3478105

[33] RitcheyER, BonginiRE, CodeKA, ZelinkaC, Petersen-JonesS, et al (2010) The pattern of expression of guanine nucleotide-binding protein beta3 in the retina is conserved across vertebrate species. Neurosci 169: 1376–1391. 10.1016/j.neuroscience.2010.05.081 20538044PMC2914127

[34] ThulinCD, HowesK, DriscollCD, SavageJR, RandTA, et al (1999) The immunolocalization and divergent roles of phosducin and phosducin-like protein in the retina. Mol Vis 5: 40 10617777

[35] CalvertPD, KrasnoperovaNV, LyubarskyAL, IsayamaT, NicoloM, et al (2000) Phototransduction in transgenic mice after targeted deletion of the rod transducin alpha-subunit. Proc Natl Acad Sci U S A 97: 13913–13918. 1109574410.1073/pnas.250478897PMC17675

[36] LyubarskyAL, NaarendorpF, ZhangX, WenselT, SimonMI, et al (2001) RGS9-1 is required for normal inactivation of mouse cone phototransduction. Mol Vis 7: 71–78. 11262419

[37] HowlettAC, GrayAJ, HunterJM, WillardsonBM (2009) Role of Molecular Chaperones in G protein β5/Regulator of G protein Signaling Dimer Assembly and G protein βγ Dimer Specificity J Biol Chem 284: 16386–16399. 10.1074/jbc.M900800200 19376773PMC2713520

[38] NikonovSS, LyubarskyA, FinaME, NikonovaES, SenguptaA, et al (2013) Cones respond to light in the absence of transducin beta subunit. J Neurosci 33: 5182–5194. 10.1523/JNEUROSCI.5204-12.2013 23516284PMC3866503

[39] KolesnikovAV, RikimaruL, HennigAK, LukasiewiczPD, FlieslerSJ, et al (2011) G-protein betagamma-complex is crucial for efficient signal amplification in vision. J Neurosci 31: 8067–8077. 10.1523/JNEUROSCI.0174-11.2011 21632928PMC3118088

[40] LobanovaES, FinkelsteinS, HerrmannR, ChenY-M, KesslerC, et al (2008) Transducin γ-subunit sets expression levels of α- and β-subunits and is crucial for rod viability. J Neurosci 28: 3510–3520. 10.1523/JNEUROSCI.0338-08.2008 18367617PMC2795350

[41] RasmussenSG, DeVreeBT, ZouY, KruseAC, ChungKY, et al (2011) Crystal structure of the beta2 adrenergic receptor-Gs protein complex. Nature 477: 549–555. 10.1038/nature10361 21772288PMC3184188

[42] LobanovaES, FinkelsteinS, SkibaNP, ArshavskyVY (2013) Proteasome overload is a common stress factor in multiple forms of inherited retinal degeneration. Proc Natl Acad Sci U S A 110: 9986–9991. 10.1073/pnas.1305521110 23716657PMC3683722

[43] WellsCA, DingusJ, HildebrandtJD (2006) Role of the chaperonin CCT/TRiC complex in G protein betagamma-dimer assembly. J Biol Chem 281: 20221–20232. 1670222310.1074/jbc.M602409200

[44] LeveillardT, Mohand-SaidS, LorentzO, HicksD, FintzAC, et al (2004) Identification and characterization of rod-derived cone viability factor. Nat Genet 36: 755–759. 1522092010.1038/ng1386

[45] PunzoC, KornackerK, CepkoCL (2009) Stimulation of the insulin/mTOR pathway delays cone death in a mouse model of retinitis pigmentosa. Nat Neurosci 12: 44–52. 10.1038/nn.2234 19060896PMC3339764

[46] GarzonJ, Rodriguez-DiazM, Lopez-FandoA, Garcia-EspanaA, Sanchez-BlazquezP (2002) Glycosylated phosducin-like protein long regulates opioid receptor function in mouse brain. Neuropharmacol 42: 813–828.10.1016/s0028-3908(02)00027-812015208

